This article has been retracted.

# Applications of Bladder Cancer Data Using a Modified Log-Logistic Model

**DOI:** 10.1155/2022/6600278

**Published:** 2022-02-02

**Authors:** Mohamed Kayid

**Affiliations:** Department of Statistics and Operations Research, College of Science, King Saud University, Riyadh, Saudi Arabia

## Abstract

In information science, modern and advanced computational methods and tools are often used to build predictive models for time-to-event data analysis. Such predictive models based on previously collected data from patients can support decision-making and prediction of clinical data. Therefore, a new simple and flexible modified log-logistic model is presented in this paper. Then, some basic statistical and reliability properties are discussed. Also, a graphical method for determining the data from the log-logistic or the proposed modified model is presented. Some methods are applied to estimate the parameters of the presented model. A simulation study is conducted to investigate the consistency and behavior of the discussed estimators. Finally, the model is fitted to two data sets and compared with some other candidates.

## 1. Introduction

In medicine, bladder cancer is the ninth most diagnosed and most common disease. There are many types and infection percentages, because among patients with bladder cancer, bladder transitional cell carcinoma accounts for about ninety percent, bladder stem cell carcinoma accounts for more than five percent, and bladder stem cell carcinoma accounts for less than two percent, depending on the pathological histology. Various lifetime models such as Rayleigh, Weibull, log-logistic, log-normal, and gamma models have been widely used to model biomedical data. Fitting a parametric model is often important for survival studies because it provides an accurate explanation of failure behavior and hazard characteristics that are not represented in nonparametric models. Some models are used in modeling lifetime experiments. An example of these models is the exponential model, which is very commonly used in life tests. In addition, there are other well-known models such as Rayleigh and Weibull. These models are still the most commonly used parameter distributions. It is well known that these models are not versatile enough to accommodate many types of data with high complexity. For almost all diseases, such as cervical, bladder, and breast cancers, the hazard rate has a unimodal or modified unimodal form.

The log-logistic (LL) model is a simple and flexible model used in survival analysis, networks, hydrology, and economics. In survival analysis, it can be used when the rate of events initially increases and later decreases, for example, in the mortality of cancer patients after diagnosis, see Bennett [1]. It has been used in networks to define the length of data transactions between applications and servers (see Gago-Benítez et al. [2]). In addition, it has been used to model channel flows and precipitation in hydrology due to its simplicity and flexible structure. See Fisk [3] for an example of how it could be used to represent the distribution of income or wealth in economics.

A well-known generalization of the LL distribution is the Burr distribution introduced by Burr [4]. Singh et al. [5] constructed a new generalized LL model for cases where the failure rate (FR) function is skewed or highly tail heavy. Ojo and Olapade [6] proposed a generalized LL distribution based on the logistic distribution and proved some properties of this distribution. Santana et al. [7] introduced a model of Kumaraswamy LL. Ramos [8] defined a new generalization of LL and discussed its properties. Gui [9] introduced a Marshall-Olkin extension of LL and studied it. Tahir et al. [10] applied the generalized beta distribution of the first kind (also called McDonald) to extend the LL distribution to a five-parameter model. Lemonte [11] defined a generalization of the beta LL generalization. Granzotto and Louzada [12] considered a transmuted LL model and studied it. Khan and Khosa [13] considered a generalized LL proportional FR model for survival data analysis. Lima and Cordeiro [14] introduced and studied an extended LL distribution with four parameters. Haghbin et al. [15] proposed a new generalized odd LL family of distributions and studied its properties. Cordeiro et al. [16] introduced a generalized odd LL family of distributions and discussed their applications. Arber and Muça [17] defined a new odd LL exponential distribution by using the generator defined by Cordeiro et al. [16]. Shakhatreh [18] applied the model of Marshal-Olking to generate an extended LL distribution. Cakmakyapan et al. [19] proposed and investigated the Kumaraswamy Marshal-Olkin LL model. Moreover, Malik and Ahmad [20] developed and studied an alpha power LL extension.

Aldahlan [21] introduced the alpha power version of LL model and studied it. Mansour [22] defined one new version of the LL model in his research. Muse et al. [23] reviewed recent research on LL distribution and its generalizations.

Muse et al. [24] applied Bayesian and classical approaches for inference about a generalized LL distribution. Alfaer et al. [25] introduced exponentiated Marshal-Olkin extension of the LL model for modeling high tail data in insurance claims.

Some of the models listed above may not be suitable for modeling a particular type of data. For example, the LL model and some of these modified versions are not appropriate when cancer patient mortality has an increasing and convex log-logistic plot (LLP), as shown in Applications. The LLP is an ascending straight line for data from the LL model, as mentioned in Subsection 2.1. Researchers are still encouraged to search for novel models in this way. Therefore, we are interested to present the modified log-logistic (MLL) model, a new and improved lifetime model. The proposed approach is highly adaptable, making it suitable for patients with bladder cancer or data from other sources with a convex and growing LLP.

This paper presents a new simple and very flexible modified version of the LL model that can describe data with decreasing, upside-down bathtub-shaped, and bathtub-shaped FR functions. The proposed model is applicable to survival analysis, networks, hydrology, economics, and many other scientific fields. The paper is organized as follows.  Section 2 presents the modified model and examines its basic statistical and reliability properties. A graphical method called LLP is presented to determine whether the data confirm the LL or the proposed MLL model.  Section 3 discusses the parameter estimation of the proposed model using six approaches, namely, the LLP method, the maximum likelihood (ML) method, the least squares (LS) method, the Anderon-Darling (AD) method, and a percentile-based (PB) method. In Section 4, a simulation study is conducted to investigate the behavior of the estimators. In Section 5, the MLL model is fitted to two data sets along with some alternatives to show the flexibility of the model. Finally, we conclude the paper in Section 6.

## 2. MLL Model

The well-known LL distribution with parameters *a* and *b*, LL(*a*, *b*), is defined by the distribution function

(1) $$\begin{array}{c} F\left(x\right)=\frac{1}{1+{\left(ax\right)}^{-b}},\;a>0,b>0,x\geq 0, \end{array}$$

and the FR function

(2) $$\begin{array}{c} \lambda \left(x\right)=\frac{ab{\left(ax\right)}^{b-1}}{1+{\left(ax\right)}^{b}}\;a>0,b>0,x\geq 0, \end{array}$$

which accommodates decreasing and upside-down bathtub-shaped FR function.

The proposed MLL model with parameters *a*, *b*, and *θ*, MLL(*a*, *b*, *θ*), is characterized by the cumulative distribution function (CDF)

(3) $$\begin{array}{c} F\left(x\right)=\frac{1}{1+{\left(ax\right)}^{-b}e^{-\theta x}},\;a>0,b>0,\theta \geq 0,x\geq 0. \end{array}$$

Then, the reliability function and the probability density function (PDF) are, respectively,

(4) $$\begin{array}{c} R\left(x\right)=\frac{1}{1+{\left(ax\right)}^{b}e^{\theta x}},\;a>0,b>0,\theta \geq 0,x\geq 0, \end{array}$$

(5) $$\begin{array}{c} f\left(x\right)=\frac{a{\left(ax\right)}^{b-1}e^{\theta x}\left(b+\theta x\right)}{{\left(1+{\left(ax\right)}^{b}e^{\theta x}\right)}^{2}},\;a>0,b>0,\theta \geq 0,x\geq 0. \end{array}$$

The PDF was plotted for some parameter values in Figure 1(a). Note that for *θ* = 0, the model reduces to the LL model.

The *p*th quantile function of MLL(*a*, *b*, *θ*), *Q*(*p*), can be obtained by solving the following equation in terms of *x*:

(6) $$\begin{array}{c} \ln\left(p^{-1}-1\right)+b\ln a=-b\ln x-\theta x. \end{array}$$

Let *Y* ~ *LL*(*a*, *b*, *θ*), and then the *k*th moment of *Y* is finite when *b* > *k*, and when *b* ≤ *k*, it is infinite. The following proposition shows that the *k*th moment of *X* ~ MLL(*a*, *b*, *θ*) is finite for almost all parameter values.

**Proposition 1 .**

For *θ* > 0, the mean of *X* ~ MLL(*a*, *b*, *θ*) is finite.

**Proof**

The mean of *X* is

(7) $$\begin{array}{c} E\left(X^{k}\right)=\int_{0}^{\infty }kx^{k-1}{\left(1+{\left(ax\right)}^{b}e^{\theta x}\right)}^{-1}dx<\int_{0}^{1}kx^{k-1}{\left(1+{\left(ax\right)}^{b}e^{\theta x}\right)}^{-1}dx+\int_{1}^{\infty }kx^{k-1}e^{-\theta x}dx<M+\frac{k}{\theta^{k}}\Gamma \left(k,\theta \right), \end{array}$$

where Γ(*k*, *θ*) is the upper incomplete gamma function. The integrand of ∫_0_^1^*kx*^*k*−1^(1 + (*ax*)^*b*^*e*^*θx*^)^−1^*dx* is a bounded and continuous function; thus, this integral is finite, and we take it to be *M*. This completes the proof.

The FR function of MLL(*a*, *b*, *θ*) is

(8) $$\begin{array}{c} \lambda \left(x\right)=a{\left(ax\right)}^{b-1}e^{\theta x}\left(b+\theta x\right)/\left(1+{\left(ax\right)}^{b}e^{\theta x}\right). \end{array}$$

Figure 1(b) shows decreasing, decreasing then increasing, and increasing then decreasing forms for the FR function.

In reliability and life testing, the concept of mean residual life (MRL) is critical. While the form of the FR function is important for repair and replacement plans, the MRL function is more important since it summarizes the entire remaining life function, whereas the first function only considers the risk of immediate failure. The MRL function of an object at time *x* indicates the mean value of the remaining life of the object given that it has survived to *x*, which can be calculated for a life model with reliability *R* as follows:

(9) $$\begin{array}{c} m\left(x\right)=\frac{1}{R\left(x\right)}\int_{x}^{\infty }R\left(t\right)dt. \end{array}$$

For the LL model, it is simplified to

(10) $$\begin{array}{c} m\left(x\right)=\left(1+{\left(ax\right)}^{b}\right)\int_{x}^{\infty }\frac{1}{1+{\left(at\right)}^{b}}dt, \end{array}$$

which is finite for *b* > 1 and infinite for *b* ≤ 1. On the other hand, for MLL(*a*, *b*, *θ*), the MRL is

(11) $$\begin{array}{c} m\left(x\right)=\left(1+{\left(ax\right)}^{b}e^{\theta x}\right)\int_{x}^{\infty }\frac{1}{1+{\left(at\right)}^{b}e^{\theta t}}dt,\;a>0,b>0,\theta >0,x\geq 0, \end{array}$$

and is finite for all parameter values, see Figure 2. However, the integral should be computed by numerical methods.

### 2.1. The LLP

From (4), we can write

(12) $$\begin{array}{c} \ln\left(\frac{1}{R\left(x\right)}-1\right)=b\ln a+b\ln x+\theta x. \end{array}$$

Taking *y* = ln((1/*R*(*x*)) − 1) and *t* = ln*x*, it simplifies to the following relation:

(13) $$\begin{array}{c} y=\beta +bt+\theta e^{t}, \end{array}$$

where *β* = *b*ln*a*. This relation shows an increasing convex curve of *y* in terms of *t*. Taking *θ* = 0, which corresponds to the LL distribution, (13) will represent a straight line.

Let *x*_1_, *x*_2_, ⋯, *x*_*n*_ be a realization from the MLL model. In an elementary but useful discrimination analysis, we can plot $y_{i}=\ln\left({\hat{R}}^{-1}\left(x_{i}\right)-1\right)$ versus *t*_*i*_ = ln*x*_*i*_, *i* = 1, 2, ⋯, *n*, called LLP. An increasing convex LLP will be in favor of the MLL while a straight line will be a clue of the LL model.  Figure 3 draws $y_{i}=\ln\left({\hat{R}}^{-1}\left(x_{i}\right)-1\right)$ versus *t*_*i*_ = ln*x*_*i*_ for three simulated samples from MLL(*a*, *b*, *θ*) with size 150 and shows how the plot diverges from the assuming straight line for different *θ*s.

## 3. Estimation of the Parameters

Suppose that *x*_1_ ≤ *x*_2_ ≤ ⋯≤*x*_*n*_ is an ordered independent and identically distributed sample from MLL(*a*, *b*, *θ*), in this section, we discuss some methods for estimating the parameters.

### 3.1. The LLP Method

This method applies the relation (13). Thus, the data are transformed into $y_{i}=\ln\left({\hat{R}}^{-1}\left(x_{i}\right)-1\right)$ and *t*_*i*_ = ln*x*_*i*_, *i* = 1, 2, ⋯, *n* where $\hat{R}\left(x\right)=n^{-1}\sum_{j=1}^{n}I\left(x_{i}>x\right)$ is the empirical reliability function. To estimate the parameters, the converted data should be fitted to the following regression model:

(14) $$\begin{array}{c} y_{i}=\beta +bt_{i}+\theta e^{t_{i}}+\epsilon_{i},\;i=1,2,\cdots ,n. \end{array}$$

The error terms *ϵ*_*i*_*s* are usually assumed to be identically distributed and independent of *N*(0, *σ*^2^). However, this assumption does not affect the estimates but is important for hypothesis tests of the parameters.

### 3.2. The ML Method

To estimate the parameters using the ML method, the following log-likelihood function should be maximized:

(15) $$\begin{array}{c} l\left(a,b,\theta ;x\right)=nb\ln a+\left(b-1\right)\overset{n}{\underset{i=1}{\sum }}\ln x_{i}+\theta \overset{n}{\underset{i=1}{\sum }}x_{i}+\overset{n}{\underset{i=1}{\sum }}\ln\left(b+\theta x_{i}\right)-2\overset{n}{\underset{i=1}{\sum }}\ln\left(1+{\left(ax_{i}\right)}^{b}e^{\theta x_{i}}\right). \end{array}$$

This expression can be maximized directly by numerical methods. In another approach, the following likelihood equations could be solved simultaneously with respect to *a*, *b*, and *θ*:

(16) $$\begin{array}{c} \frac{\partial }{\partial a}l\left(a,b,\theta ;x\right)=\frac{nb}{a}-2\overset{n}{\underset{i=1}{\sum }}\frac{b{\left(ax_{i}\right)}^{b-1}x_{i}e^{\theta x_{i}}}{1+{\left(ax_{i}\right)}^{b}e^{\theta {\text{x}}_{i}}}=0,\\ \frac{\partial }{\partial b}l\left(a,b,\theta ;x\right)=n\ln a+\overset{n}{\underset{i=1}{\sum }}\ln x_{i}+\overset{n}{\underset{i=1}{\sum }}\frac{1}{b+\theta x_{i}}-2\overset{n}{\underset{i=1}{\sum }}\frac{\ln\left(ax_{i}\right){\left(ax_{i}\right)}^{b}e^{\theta x_{i}}}{1+{\left(ax_{i}\right)}^{b}e^{\theta x_{i}}}=0,\\ \frac{\partial }{\partial \theta }l\left(a,b,\theta ;x\right)=\overset{n}{\underset{i=1}{\sum }}x_{i}+\overset{n}{\underset{i=1}{\sum }}\frac{x_{i}}{b+\theta x_{i}}-2\overset{n}{\underset{i=1}{\sum }}\frac{{\left(ax_{i}\right)}^{b}x_{i}e^{\theta x_{i}}}{1+{\left(ax_{i}\right)}^{b}e^{\theta x_{i}}}=0. \end{array}$$

The Fisher information matrix is of the form

(17) $$\begin{array}{c} K=\left[\begin{array}{ccc} E\left(-\frac{\partial^{2}l}{\partial a^{2}}\right) & E\left(-\frac{\partial^{2}l}{\partial a\partial b}\right) & E\left(-\frac{\partial^{2}l}{\partial a\partial \theta }\right)\\ E\left(-\frac{\partial^{2}l}{\partial b\partial a}\right) & E\left(-\frac{\partial^{2}l}{\partial b^{2}}\right) & E\left(-\frac{\partial^{2}l}{\partial b\partial \theta }\right)\\ E\left(-\frac{\partial^{2}l}{\partial \theta \partial a}\right) & E\left(-\frac{\partial^{2}l}{\partial \theta \partial b}\right) & E\left(-\frac{\partial^{2}l}{\partial \theta^{2}}\right) \end{array}\right], \end{array}$$

where *l* = ln*f*(*X*) represents the log-likelihood function. The variance-covariance matrix of the MLE can be approximated by *n*^−1^*K*^−1^, where *K*^−1^ is the inverse of the information matrix. Moreover, for a coefficient matrix *A* such that *K*^−1^ = *AA*^*T*^, the random vector

(18) $$\begin{array}{c} \sqrt{n}A\left(\hat{a}-a,\hat{b}-b,\hat{\theta }-\theta \right), \end{array}$$

converges vaguely to a standard normal random vector.

### 3.3. The MPS Method

In this approach, the following spaces are considered.

(19) $$\begin{array}{c} D_{i}=F\left(x_{i}\right)-F\left(x_{i-1}\right),\;\;\;i=1,2,\cdots ,n+1, \end{array}$$

where *x*_0_ = 0 and *x*_*n*+1_ = ∞. Then, the logarithm of product spacing function

(20) $$\begin{array}{c} l_{p}\left(a,b,\theta ;x\right)=\overset{n+1}{\underset{i=1}{\sum }}\ln D_{i}, \end{array}$$

is maximized subject to (*a*, *b*, *θ*) to find the estimates of the parameters. This method was proposed by Cheng and Amin [26], and they have shown its efficiency. Here, *l*_*p*_(*a*, *b*, *θ*; *x*) reduces to

(21) $$\begin{array}{c} l_{p}\left(a,b,\theta ;x\right)=\ln\left(1-\frac{1}{1+{\left(ax_{1}\right)}^{b}e^{\theta x_{1}}}\right)+\ln\left(\frac{1}{1+{\left(ax_{n}\right)}^{b}e^{\theta x_{n}}}\right)+\overset{n}{\underset{i=2}{\sum }}\ln\left(\frac{1}{1+{\left(ax_{i-1}\right)}^{b}e^{\theta x_{i-1}}}-\frac{1}{1+{\left(ax_{i}\right)}^{b}e^{\theta x_{i}}}\right). \end{array}$$

### 3.4. The LS Method

In the least squares method, the estimates of the parameters are computed by minimizing sum of the squared distances between the estimated and the empirical distribution functions, i.e.,

(22) $$\begin{array}{c} \left(\hat{a},\hat{b},\hat{\theta }\right)=\arg\underset{a,b,\theta }{\min}\;\overset{n}{\underset{i=1}{\sum }}{\left(\frac{1}{1+{\left(ax_{i}\right)}^{\text{b}}e^{\theta x_{i}}}-\frac{n-i+1}{n+1}\right)}^{2}. \end{array}$$

This method is also called Cramer-von Mises.

### 3.5. The AD Method

To estimate the parameters using the method AD, we should minimize sum of the weighted squared distances between the estimated and the empirical distribution function, i.e.,

(23) $$\begin{array}{c} \overset{n}{\underset{i=1}{\sum }}\frac{1}{F\left(x_{i}\right)\left(1-F\left(x_{i}\right)\right)}{\left(F\left(x_{i}\right)-\hat{F}\left(x_{i}\right)\right)}^{2}, \end{array}$$

where $\hat{F}\left(x_{i}\right)$ shows the empirical distribution function at point *x*_*i*_. Thus, for MLL, the AD estimates are computed by the following relation:

(24) $$\begin{array}{c} \left(\hat{a},\hat{b},\hat{\theta }\right)=\arg\underset{a,b,\theta }{\min}\;\overset{n}{\underset{i=1}{\sum }}\left(1+{\left(ax_{i}\right)}^{b}e^{\theta x_{i}}\right)\times \left(1+{\left(ax_{i}\right)}^{-b}e^{-\theta x_{i}}\right){\left(\frac{1}{1+{\left(ax_{i}\right)}^{b}e^{\theta x_{i}}}-\frac{n-i+1}{n+1}\right)}^{2}. \end{array}$$

### 3.6. The PB Method

The PB estimates of the parameters can be computed by minimizing sum of the squared distances between the estimated and empirical quantiles. By taking the observation *x*_*i*_ as the empirical *i*/(*n* + 1)th quantile, we could estimate the parameters by

(25) $$\begin{array}{c} \left(\hat{a},\hat{b},\hat{\theta }\right)=\arg\underset{a,b,\theta }{\min}\;\overset{n}{\underset{i=1}{\sum }}{\left(Q\left(\frac{i}{n+1}\right)-x_{i}\right)}^{2}, \end{array}$$

where *Q*(*p*) is the *p*th quantile function of MLL(*a*, *b*, *θ*), defined in (6), and depends on (*a*, *b*, *θ*).

## 4. Simulations

To generate a random sample from MLL(*a*, *b*, *θ*), we solve the equation *F*(*X*) = *U* with respect to *X*, where *U* is a generated instance from the standard uniform distribution. The answer for *X* is the square root of the function

(26) $$\begin{array}{c} g\left(X\right)=b\ln X+\theta X-c, \end{array}$$

where *c* = ln(*U*^−1^ − 1) + *b*ln*a*. From the fact that *g* is strictly increasing, lim_*x*⟶0^+^_*g*(*x*) = −∞ and *g*(1) = *θ* − *c*, we can conclude that if *θ* < *c*, then *X* > 1 and if *θ* ≥ *c*, then *X* ≤ 1. Thus, we can restrict range of the correct answers for *X* based on the parameters. In each run, *r* = 5000 replicates of random samples are extracted from the MLL distribution with selected parameters.

The samples are of size *n* = 50, 100, or 200, and then, the estimates ML, LLP, LS, PB, MPS, or AD are calculated for each sample. The optimization to compute the ML, LS, PB, AD, and MPS estimates is performed by the “optim” function using the standard “Nelder-Mead” method in R. The initial values needed to maximize or minimize the objective functions are randomly derived from the uniform model, e.g., for *a* on the intervals *a* × (0.85,1.25) and similarly for *b* and *θ*. For the LLP method, the built-in function “lm” in R is used. The results are summarized in Tables 1–3. Each cell in these tables shows the results for one run and gives the bias (*B*) and mean square error (MSE) for all parameters.

Some important observations from the simulation results listed in Tables 1–3 are given below:

- The values of *B* and MSE decrease with *n*, indicating that all estimators considered are consistent
- The small values of *B* and MSE show that all considered methods are suitable for application in real problems
- The PB estimator performs better than all others in terms of MSE. The second best results are related to the AD estimator. The ML and MPS estimators show similar results

## 5. Applications

In this section, we fit the proposed model to two data sets and present some possible alternatives. According to Al-Shomrani et al. [27], the first data set contains the remission times (in months) for 128 patients with bladder cancer, which are shown in Table 4.  Figure 4(a) shows a unimodal (upside-down bathtub shape) FR function for the data in the Total Time on Test (TTT) plot. In addition, the LLP in Figure 4(b) shows a convex curve that obviously favors the MLL model.

The alternative models considered here are the generalized gamma (GG), LL, Marshal-Olkin log-logistic (MOLL), exponentiated Weibull (EW), beta LL (BLL), and Kumaraswamy LL (KLL) with the CDFs or PDFs, respectively

(27) $$\begin{array}{c} F\left(x\right)=1-\frac{\Gamma \left(b,{\left(ax\right)}^{\theta }\right)\;}{\Gamma \left(b\right)},\;a>0,b>0,x\geq 0,\\ F\left(x\right)=\frac{1}{1+{\left(ax\right)}^{b}},\;a>0,b>0,x\geq 0,\\ F\left(x\right)=\frac{\theta {\left(1+{\left(ax\right)}^{b}\right)}^{-1}}{1-\left(1-\theta \right){\left(1+{\left(ax\right)}^{b}\right)}^{-1}},\;a>0,b>0,\theta >0,x\geq 0,\\ F\left(x\right)={\left(1-\exp\left(-ax^{b}\right)\right)}^{\theta },\;a>0,b>0,\theta >0,x\geq 0,\\ f\left(x\right)=\frac{1}{B\left(a,b\right)}\frac{\alpha }{\beta }{\left(\frac{x}{\beta }\right)}^{a\alpha -1}{\left(1+{\left(\frac{x}{\beta }\right)}^{\alpha }\right)}^{-a-b},\;a>0,b>0,\alpha >0,\beta >0,x\geq 0,\\ f\left(x\right)=ab\;\frac{\alpha }{\beta }{\left(\frac{x}{\beta }\right)}^{a\alpha -1}{\left(1+{\left(\frac{x}{\beta }\right)}^{\alpha }\right)}^{-a-1}{\left[1-{\left\{1-{\left(1+{\left(\frac{x}{\beta }\right)}^{\alpha }\right)}^{-1}\right\}}^{a}\right]}^{b-1},\;a>0,b>0,\alpha >0,\beta >0,x\geq 0, \end{array}$$

where Γ(*b*, *y*) = ∫_*y*_^∞^*t*^*b*−1^*e*^−*t*^*dt* is the upper incomplete gamma function.

Tahir et al. [10] studied the BLL and KLL. The “optim” function uses the usual “Nelder-Mead” approach in R to compute the ML estimates of the parameters for all selected models. Moreover, the AIC, Kolmogorov–Smirnov (K-S), AD, and Cramer-Von Mises (CVM) statistics are computed.  Table 5 summarizes the results and shows that the MLL outperforms other models in terms of all computed statistics, however, in a close competition.  Figure 5 shows the empirical and estimated distribution functions of the selected models.

The second data set, shown in Table 6, represents the number of claims from private motor insurance policies in the United Kingdom studied by Alfaer et al. [25]. The TTT graph is plotted in Figure 6(a) and shows a decreasing FR function. The LLP is plotted in Figure 6(b) and shows a convex curve. The results of fitting the MLL model and all alternatives considered are summarized in Table 7. The results show that the MLL model provides a better description of the data than all other models considered.  Figure 7 presents the CDF of the estimated models and the empirical CDF for graphical examination.

## 6. Conclusion

The proposed MLL model presented in this paper can be useful in many situations where the FR function has a bathtub shape, an upside-down bathtub shape, or a decreasing shape and in the case when the LLP exhibits an increasing and convex curve. To estimate the parameters, LLP, ML, MPS, LS, AD, and PB methods are discussed. Simulation results show that all methods provide consistent estimators and give sufficiently accurate estimates of the parameters. The model is fitted to two data sets and compared with some other candidates. In terms of all calculated statistics, the MLL model outperforms the other models for the first data set. In addition, the MLL model provides a better description of the second data set than all other models considered.

## Figures and Tables

**Figure 1:** The PDF (a) and the FR function (b) of the MLL for some parameter values.

**Figure 2:** The MRL (a) and the median residual life function (b) of the MLL for some parameter values.

**Figure 3:** The LLP for three simulated samples from the MLL model. The straight line shows the corresponding LLP of the LL model.

**Figure 4:** The TTT plot (a) and LLP (b) for data set of Table 4.

**Figure 5:** The empirical distribution function of remission times along with estimated models.

**Figure 6:** The TTT plot (a) and LLP (b) for data set of Table 6.

**Figure 7:** The empirical distribution function of loss data (Table 6) along with estimated models.

**Table 1:** The bias and MSE of the ML and LLP estimators computed by a simulation study. Each cell consists of *B*_*a*_ and MSE_*a*_ in the first row, *B*_*b*_ and MSE_*b*_ in the second row, and *B*_*θ*_ and MSE_*θ*_ in the third row.

		*n*					
Method	*a*, *b*, *θ*	50		100		200	
		*B*	MSE	*B*	MSE	*B*	MSE
ML	0.1, 1.5, 0.01	-0.0149	0.0014	-0.0116	0.0011	-0.0088	0.0008
		-0.1754	0.2413	-0.1397	0.1921	-0.1111	0.1486
		0.0188	0.0018	0.0128	0.0011	0.0090	0.0007
	0.1, 0.8, 0.03	-0.0001	0.0017	-0.0012	0.0008	6.3 × 10^−6^	0.0004
		0.0037	0.0312	-0.0011	0.0154	0.0005	0.0092
		0.0044	0.0003	0.0022	0.0001	0.0011	7.2 × 10^−5^
	0.3, 1.2, 0.02	-0.0153	0.0052	-0.0063	0.0025	-0.0032	0.0012
		-0.0271	0.0379	-0.0140	0.0185	-0.0060	0.0092
		0.0170	0.0014	0.0080	0.0005	0.0040	0.0002
	0.3, 0.7, 0.08	0.0134	0.0193	0.0018	0.0087	0.0013	0.0042
		0.0148	0.0207	0.0045	0.0093	0.0031	0.0046
		0.0075	0.0015	0.0047	0.0007	0.0019	0.0003
LLP	0.1, 1.5, 0.01	-0.0105	0.0008	-0.0069	0.0004	-0.0042	0.0002
		-0.1673	0.1275	-0.1144	0.0624	-0.0768	0.0285
		0.0164	0.0009	0.0098	0.0003	0.0057	0.0001
	0.1, 0.8, 0.03	-0.0066	0.0019	-0.0076	0.0010	-0.0050	0.0004
		-0.0790	0.0351	-0.0608	0.0182	-0.0375	0.0087
		0.0106	0.0005	0.0069	0.0002	0.0041	8.2×10^−5^
	0.3, 1.2, 0.02	0.0213	0.0078	-0.0119	0.0032	-0.0072	0.0014
		-0.1245	0.0672	-0.0808	0.0312	-0.0493	0.0144
		0.0318	0.0035	0.0166	0.0010	0.0093	0.0003
	0.3, 0.7, 0.08	-0.0094	0.0220	-0.0128	0.0103	-0.0121	0.0048
		-0.0611	0.0247	-0.0460	0.0126	-0.0300	0.0061
		0.0252	0.0028	0.0158	0.0011	0.0091	0.0005

**Table 2:** The bias and MSE of the LS and AD estimators computed by a simulation study. Each cell consists of *B*_*a*_ and MSE_*a*_ in the first row, *B*_*b*_ and MSE_*b*_ in the second row, and *B*_*θ*_ and MSE_*θ*_ in the third row.

		*n*					
Method	*a*, *b*, *θ*	50		100		200	
		*B*	MSE	*B*	MSE	*B*	MSE
LS	0.1, 1.5, 0.01	-0.0078	0.0008	-0.0045	0.00041	-0.0022	0.00019
		-0.1071	0.1128	-0.0589	0.0592	-0.0290	0.0298
		0.0105	0.0009	0.0085	0.00039	0.0027	0.00018
	0.1, 0.8, 0.03	0.0021	0.0022	-0.00002	0.00107	0.0012	0.00054
		-0.0110	0.0426	-0.0075	0.0211	0.00005	0.0103
		0.0019	0.0005	0.0008	0.0002	0.00006	0.0001
	0.3, 1.2, 0.02	-0.0169	0.0073	-0.0069	0.0035	-0.0039	0.0017
		-0.0663	0.0600	-0.0345	0.0288	-0.0156	0.0153
		0.0189	0.0032	0.0087	0.0012	0.0046	0.00057
	0.3, 0.7, 0.08	0.0176	0.0250	0.0044	0.0111	0.0019	0.0053
		-0.0075	0.0310	-0.0043	0.0145	-0.0029	0.0069
		0.0032	0.0027	0.0022	0.0013	0.0009	0.00059
AD	0.1, 1.5, 0.01	-0.0027	0.00051	-0.00095	0.00025	0.00018	0.00011
		-0.1102	0.0707	-0.0519	0.0385	-0.0195	0.0188
		0.0034	0.00032	0.0012	0.00015	-0.00017	0.00007
	0.1, 0.8, 0.03	0.0046	0.0019	0.0017	0.00087	0.0022	0.00044
		-0.0335	0.0283	-0.0201	0.0141	-0.0056	0.00696
		-0.0009	0.00025	-0.0008	0.00012	-0.0008	0.00006
	0.3, 1.2, 0.02	-0.0045	0.0053	0.0018	0.0026	0.0023	0.0012
		-0.0820	0.0417	-0.0357	0.0201	-0.0115	0.0102
		0.0060	0.0011	0.0005	0.00043	-0.0009	0.00021
	0.3, 0.7, 0.08	0.0260	0.0224	0.0102	0.0096	0.0065	0.0045
		-0.0262	0.0213	-0.0149	0.0097	-0.0057	0.0049
		-0.0044	0.0015	-0.0024	0.00071	-0.0021	0.00035

**Table 3:** The bias and MSE of the PB and MPS computed by a simulation study. Every cell consists of *B*_*a*_ and MSE_*a*_ in the first row, *B*_*b*_ and MSE_*b*_ in the second row, and *B*_*θ*_ and MSE_*θ*_ in the third row.

		*n*					
Method	*a*, *b*, *θ*	50		100		200	
		*B*	MSE	*B*	MSE	*B*	MSE
PB	0.1, 1.5, 0.01	-0.0013	6.44 × 10^−5^	-0.0012	6.41 × 10^−5^	-0.0012	6.38 × 10^−5^
		-0.0185	0.0144	-0.0186	0.0143	-0.0189	0.0139
		-0.00010	6.55 × 10^−7^	-0.00011	6.54 × 10^−7^	-0.00012	6.43 × 10^−7^
	0.1, 0.8, 0.03	-0.0015	6.52 × 10^−5^	-0.0010	6.43 × 10^−5^	-0.0014	6.36 × 10^−5^
		-0.0089	0.0042	-0.0105	0.0040	-0.0112	0.0039
		-0.0004	5.91 × 10^−6^	-0.0004	5.86 × 10^−6^	-0.0003	5.77 × 10^−6^
	0.3, 1.2, 0.02	-0.0041	0.00058	-0.00038	0.00057	-0.0040	0.0057
		-0.0138	0.0093	-0.0127	0.0092	-0.0167	0.0091
		0.0002	2.58 × 10^−6^	-0.0002	2.56 × 10^−6^	-0.0002	2.52 × 10^−6^
	0.3, 0.7, 0.08	-0.0035	0.00057	-0.0039	0.00056	-0.0037	0.00054
		-0.0072	0.0032	-0.0097	0.0031	-0.0084	0.0031
		-0.0008	4.04 × 10^−5^	-0.0008	4.01 × 10^−5^	-0.0010	4.01 × 10^−5^
MPS	0.1, 1.5, 0.01	-0.0023	0.0005	-0.0006	0.00024	0.0005	0.0001
		-0.0829	0.0657	-0.0371	0.0359	-0.0122	0.0172
		0.0032	0.00031	0.0008	0.00013	-0.00053	6.07 × 10^−5^
	0.1, 0.8, 0.03	0.0046	0.0018	0.0027	0.00084	0.0020	0.00042
		-0.0202	0.0277	-0.0097	0.0134	-0.0057	0.0068
		-0.0006	0.00025	-0.0010	0.00011	-0.0007	5.52 × 10^−5^
	0.3, 1.2, 0.02	-0.0016	0.0054	0.0026	0.0025	0.0024	0.0012
		-0.0565	0.0373	-0.0211	0.0185	-0.0088	0.0092
		0.0047	0.0010	-0.0005	0.0003	-0.0011	0.00018
	0.3, 0.7, 0.08	0.0304	0.0173	0.0236	0.0093	0.0136	0.0045
		0.0880	0.0312	0.0544	0.0136	0.0306	0.0059
		-0.0155	0.0015	-0.0108	0.0007	-0.0067	0.00035

**Table 4:** Remission times (in month) of bladder cancer for 128 patients.

0.08	2.09	3.48	4.87	6.94	8.66	13.11	23.63	0.20	2.23
3.52	4.98	6.97	9.02	13.29	0.40	2.26	3.57	5.06	7.09
9.22	13.80	25.74	0.50	2.46	3.64	5.09	7.26	9.47	14.24
25.82	0.51	2.54	3.70	5.17	7.28	9.74	14.76	26.31	0.81
2.62	3.82	5.32	7.32	10.06	14.77	32.15	2.64	3.88	5.32
7.39	10.34	14.83	34.26	0.90	2.69	4.18	5.34	7.59	0.66
15.96	36.66	1.05	2.69	4.23	5.41	7.62	10.75	16.62	43.01
1.19	2.75	4.26	5.41	7.63	17.12	46.12	1.26	2.83	4.33
5.49	7.66	11.25	17.14	79.05	1.35	2.87	5.62	7.87	11.64
17.36	1.40	3.02	4.34	5.71	7.93	11.79	18.10	1.46	4.40
5.85	8.26	11.98	19.13	1.76	3.25	4.50	6.25	8.37	12.02
2.02	3.31	4.51	6.54	8.53	12.03	20.28	2.02	3.36	6.76
12.07	21.73	2.07	3.36	6.93	8.65	12.63	22.69		

**Table 5:** Results of fitting MLL and some alternative models to data set of Table 4.

Model	$\hat{a}$	$\hat{b}$	$\hat{\theta }$ $\left(\hat{\alpha }\right)$	$\hat{\beta }$	AIC	K-S *P* value	AD *P* value	CVM *P* value
MLL	0.1391	1.4215	0.0358	—	823.99	0.0331 0.9990	0.1258 0.9997	0.0185 0.9982
GG	1.6986	3.6989	0.5159	—	826.12	0.0463 0.9462	0.2841 0.9495	0.0452 0.9053
LL	0.1674	1.6945	—	—	825.77	0.0392 0.9893	0.2684 0.9597	0.0223 0.9944
MOLL	0.1004	1.6944	0.4202	—	827.77	0.0393 0.9889	0.2685 0.9596	0.0224 0.9943
EW	2.5485	0.2577	34.81	—	847.78	0.0846 0.3186	1.4773 0.1820	0.2486 0.1902
BLL	0.6992	1.3529	1.8257	10.4444	826.00	0.0338 0.9986	0.1155 0.9999	0.0196 0.9974
KLL	3.7385	20.2571	0.4967	13.5393	827.29	0.0426 0.9741	0.2163 0.9853	0.0334 0.9642

**Table 6:** The number of claims of losses from private passenger automobile insurance policies in United Kingdom.

21	40	23	5	63	171	92	44	140	343
318	129	123	448	361	169	151	479	381	166
245	970	719	304	266	859	504	162	260	578
312	96								

**Table 7:** Results of fitting MLL and some alternative models to data set of Table 6.

Model	$\hat{a}$	$\hat{b}$	$\hat{\theta }$ $\left(\hat{\alpha }\right)$	$\hat{\beta }$	AIC	K-S *P* value	AD *P* value	CVM *P* value
MLL	0.0033	1.2730	0.0021	—	430.65	0.0847 0.9606	0.2227 0.9829	0.0287 0.9817
GG	0.1911	5.0856	0.4336	—	432.02	0.0957 0.9038	0.3350 0.9091	0.0525 0.8643
LL	0.0051	1.6014	—	—	432.76	0.0870 0.9513	0.4383 0.8089	0.0481 0.8905
MOLL	0.0043	1.6014	0.7701	—	434.76	0.0872 0.9504	0.4383 0.8089	0.0482 0.8899
EW	0.9916	0.2573	27.3839	—	440.27	0.1528 0.4025	0.8930 0.4177	0.1586 0.3657
BLL	9.9905	13.8848	0.3795	430.48	437.25	0.1226 0.6762	0.6067 0.6403	0.1003 0.5864
KLL	36.1320	20.2882	0.3143	0.1132	436.64	0.1159 0.7394	0.5322 0.7129	0.0847 0.6683

## Data Availability

The data used to support the findings of this study are included within the article.
